The article "An Overview of the Implications for Perianesthesia Nurses in terms of Intraoperative Changes in Temperature and Factors Associated with Unintentional Postoperative Hypothermia" was published in 2022. Journal: J Healthc Eng.

# An Overview of the Implications for Perianesthesia Nurses in terms of Intraoperative Changes in Temperature and Factors Associated with Unintentional Postoperative Hypothermia

**DOI:** 10.1155/2022/6955870

**Published:** 2022-04-11

**Authors:** Fang Yang, Jing Wang, Jifang Cui, Jia Zhuan, Xiaoyan Hu, Shuting Chen

**Affiliations:** Clean Operation Department, Qinghai People's Hospital, Qinghai 810000, China

## Abstract

Patients undergo surgery and anaesthesia on a daily basis across the United States and throughout the world. A major source of worry for these patients continues to be inadvertent hypothermia, once core temperature <36°C (96.8°F). Despite well-documented adverse physiological consequences, anaesthesia nurses continue to have a difficult task in keeping patient warmth pre-/peri-/post-surgical procedure. Thermostasis within postoperative patient necessitates the collaboration of many individuals. In order to provide safe and high-quality treatment, it is essential to use the most up-to-date data to guide therapeutic procedures targeted at achieving balance body temperature in surgical patients. Providing a review of the physiology of perioperative temperature variations and the comorbidities linked with accidental intraoperative hypothermia, this article will also provide preventive and treatment methods.

## 1. Introduction

Patients undergoing surgery and anaesthesia often experience drops in core-body temperature to <36°C (96.8°F) [1–3]. Hypothermia is characterised by widespread metabolism reduction that affects all bodily systems at the same time. Between 50 and 90 percent of surgery patients suffer from hypothermia at some point throughout their recovery period [4, 5]. The consequence is significant physiological alterations, including changed heart function, fluctuations in state of awareness, shivering and extended plasma half-lives of medicines, which may also enhance oxygen consumption by up to 500 percent [6–8]. Hypothermia is linked with a number of additional negative outcomes, including an increase in the duration of hospital stay, an increase in infection rates, and an increase in cardiac events [9]. According to research, individuals who maintain a normal body temperature during the surgical process are less likely to get infections (64 percent), have 44 percent less cardiac problems, and are 34 percent fewer likely to need perioperative mechanical breathing. Furthermore, patients who got hypothermic were discharged from the hospital 40 percent sooner than those who did not become hypothermic [9, 10]. A solid understanding of the factors that contribute to perioperative hypothermia, as well as the mechanism of heat exchange in operating patients during their perianesthesia and post-surgical time frame, and also the physiologic changes related with this heat loss, are required for the implementation of guiding principles in the perianesthesia context [11]. It is also necessary to be familiar with the risk factors for hypothermia. Perianesthesia nurses continue to play a significant role in maintaining thermal balance in surgical patients. In the postoperative care of operating patients, via treatments targeted at reducing temperature loss, however preserving and/or recovering normothermia differentiates the difficulty faced by perianesthesia nurses from other types of challenges [11–13].

Herein, we first explained the temperature monitoring for patient undergoing anaesthesia and the basic science and temperature regulation physiology of heat lost from a patient to the environment. We explained the various risk factors to improve intraoperative heat control throughout the process. Next, we highlight the perianesthetic heat loss and the phenomena, balance between thermolysis and thermogenesis and the physiological changes as a result of hypothermia, as well as the various variables for the improvement of perioperative hypothermia. Finally, we highlight the hypothermia and its consequences and provide the concluding remarks. This review will give readers an overview of the implications for perianesthesia nurses in terms of intraoperative changes in temperature and factors associated for unintentional post-operative hypothermia.

## 2. Temperature Monitoring

“Every patient undergoing anaesthesia should have his or her temperature monitored whenever clinically significant changes in body temperature are intended, expected, or suspected,” as described by the American Society of Anesthesiologists' guidelines concerning fundamental anaesthetic observation [14]. Due to the fact that this recommendation does not specify the method of temperature monitoring to be used, when to monitor, or for how long to monitor, variability in patient safety and broad variance in clinical practise will result. The American Society of Perianesthesia Nurses (ASPAN) recommendations offer scientific proof guidelines for monitoring temperature in anaesthesia care settings[15].

Inner abdominal-area / thorax /neural tissue-temperature is defined as CT (CT). This temperature is carefully regulated, and it is typically 2 – 4°C (3.6 – 7.2 degrees Fahrenheit) elevated in comparison to dermal thermo-readings. During general anaesthesia, CTs remain frequently monitored across several sites such as the distal oesophagus, bladder (in instances of excessive urine flow), nasopharynx, and the pulmonary artery, among other places. The CT of people is the single greatest indication of their thermal state, despite the fact that it is not fully representative of their body heat content and distribution [16]. Axillary, rectal, bladder (having low urine flow), and mouth measures of near-CTs are more frequently utilised in regional anaesthetic patients during the perioperative period than other methods of temperature monitoring. This kind of measurement is usually less difficult to acquire, although it is influenced by external factors (such as the surrounding environment's temperature) and internal factors (such as the body's regional cutaneous blood flow). When it comes to axillary and oral temperatures, this concept makes sense, but the differences between bladder and rectal temperatures are less apparent. Temperatures in the rectal area are usually very closely related to CTs [17–19]. In the event of malignant hyperthermia (MH) and heat stroke, however, these precautions are not taken [20–22]. Furthermore, because rectal temperature lags after true CT during cardiac bypass, it is considered a near CT in patients who have been deliberately chilled. As a result, while taking rectal temperature readings, extreme care must be used. When urine flow is high, bladder temperature equals pulmonary artery thermal-reading / CT; however, upon reduced urine output, bladder temperature come close to rectal temperature [23, 24]. Beside this, temperature of bladder is also regarded to be a near-core metric because of its reliance on urine flow. As a result, the capacity of any of these measurements to represent CT is severely restricted. The most appropriate thermoregulatory monitoring location throughout periperative, intra-operative and after operation timeframes remains disputed, with the best source varying depending on the age of the patient. Preoperative temperature measures are most frequently taken by mouth for adults, oral or axillary temperature measurements are taken by mouth for paediatric patients, and axillary measurements are taken by hand for newborns. When feasible, an esophageal probes are employed for intra-surgical patient CT determinations. This technique is relatively safe / inexpensive, offering peak precise evaluation for thermo-readings available on the market. Furthermore, this measurement is the most precise when there are significant fluctuations in temperature. However, measuring the oesophagus is more difficult in patients receiving regional or controlled anaesthesia, as well as in those who are recovering from surgery. Except in the case of severe thermal disturbances, CTs may be calculated with acceptable precision from near-core observations taken near the core [25–27]. The application of a liquid-crystal temperature strip to the forehead is another popular method of thermal monitoring. These gadgets are low-cost, non-invasive, and simple to use, making them an excellent choice. Despite the fact that dermal thermo-reading remain significantly lesser in comparison to CT-readings, with increased vulnerability to environmental temperatures, these strips will offer a good approximation of CTs when regulated with a proper off-set (0.5uC in conscious individuals, 1uC in drowsy/anesthetized individuals) [28]. 19 When temperature fluctuations are more severe, for as during MH, liquid-crystal thermal-strips prove ineffective for noticing temperature rises within porcine models [29]. Such detectors were un-evaluated in people regarding this role, consequently not being recommended for human MH determination [30] . As a result of these considerations, CTs / near-CTs could become employed within the peri-surgical timeframes once risk-benefit analyses are concluded, knowing that clinical-setting situations could necessitate the use of a different technique.

The new AORN “Guideline for prevention of unintended patient hypothermia” gives guidelines in recognizing parameters related to intra-surgical hypothermia and its circumvention, teaching peri-surgical professionals regarding this issue, together with implementing applicable guidelines / protocols (Figure 1) [31].

## 3. Background Basic Science

There are four different ways through which heat may be lost from a patient to the environment. Radiation and convection are the most significant contributions to global warming [32]. Heat is emitted by any surfaces that are warmer than absolute zero, which is known as radiation (thermal) (infrared radiation). This emitted heat is absorbed by all surfaces in the immediate vicinity. As a result, the patient generates heat that is radiated into the surrounding environment. During surgery, radiation is most likely the most significant heat-loss source.

### 3.1. Convection

Usually, minute layers of static-air in proximity to the dermal layer serve as insulation, preventing conduction-based heat from being transmitted through the skin to nearby air molecules. Once air currents pass across it, this layer is disturbed, the insulating qualities of the layer are significantly reduced, resulting in increased heat loss. Convection is the term used to describe this process, which is the foundation for the notion of wind cold factor. When it comes to non-OR hospital settings, room air is usually replaced four times per hour, whereas in distinctive operating room (OR), room air is circulated fifteen times per hour. Because of the little perceptible flow of air throughout the operating room, these rooms are perceived as being cooler. Surgical curtains serve as thermal insulators, reducing convective heat loss to a bare minimum. Contrary to popular belief, convection-based heat-loss forms 2nd paramount cause for thermal-losses within OR.

### 3.2. Conduction

Conduction can be described as thermal-transference through conductive media deprived of any discernible movement of the medium itself. Because of the temperature differential between two mediums and the material's heat conductivity, heat transfer occurs at a faster pace in certain cases. For the reason that the patient is in close touch with foam protecting sheet on the operating table, conduction contributes only a small portion of the heat loss during surgery.

### 3.3. Evaporation

This can be described as transformation of liquids into vapors once temperature is below the boiling point. As a result, molecules with the greatest kinetic energy can escape from a liquid's surface, decreasing the kinetic energy (KE) and therefore reduce the temperature. This kind of thermal loss is most often seen when sterile preparation solutions are used in the manufacturing process. It is possible that evaporative losses from surgical wounds will also be a factor [32].

### 3.4. Temperature regulation physiology

The human thermoregulatory system is capable of maintaining a constant body temperature inside under typical conditions; the usual body temperature is about 37°C. In the operating room, on the other hand, a collection of changed thermoregulatory mechanisms and lower ambient temperatures classically leads a reduction in CT. Hypothermia takes place once CT is less than 36°C, is a reasonably frequent occurrence within operating patients, with a frequency of up to 20% reported. Cases occur when healthy individuals experience CT drops of 0.5 - 1.5°C [33, 34] in the first hour after undergoing a surgical operation.

Physiologic thermoregulation is comprised of a system of afferent temperature sensing, efferent reactions and central regulation that works in concert. Thermosensing cellular populations found within spinal cord, brain, thorax, skin surface together with deep abdominal tissue are responsible for afferent thermal perception in hypothermia [35]. The hypothalamus, with reduced aid by the spinal cord, are responsible for central CT regulation. Endpoints to hypothermia in adults manifests itself mainly via behavioural change, although it may also express itself through vasoconstriction and shivering. Additionally, nonshivering thermogenesis is shown in neonates, and various physiological changes are associated with the with the hypothermia (Figure 2).

### 3.5. Thermoregulation and aesthetic effects

The body's temperature is well controlled under normal conditions by controlling blood flow using arteriovenous shunts, which have been located on the surface of skin and regulate blood flow. It is possible that this blood flow accounts for as much as 10% of the total cardiac output, and that vasoconstriction might cause an improvement in mean arterial blood pressure of about 15 mmHg [36–38]. Anesthesia has a significant impact on the body's thermoregulatory systems. The use of general anaesthetics may help prevent heat loss-driven vasoconstriction, leading to improvement in patient thermal regulation once they are exposed to a frigid environment. The heat produced by the body is not dispersed evenly. Relatively, heat is often focused within core-regions, namely the head / trunk regions, with peripheral regions remaining lower in temperature. It's important to observe that heat from the core is directed towards the periphery body-stress manifests by decreasing OR temperatures / vasodilation functions through generalized anaesthetic take effect due to a lack of sympathetic tone (Figure 3) [33]. Such change leads into fast CT drop, approximating 0.5-1.5°C (0.9–2.7°F), which may be detected within the first hour after surgery. As a consequence of the vasodilation characteristics of general anaesthetics, this redistribution hypothermia is not a true loss of heat, but instead of a transfer in heat energy from the central to the periphery, which causes the patient to become hypothermic. Following the administration of general anaesthesia, the warmer periphery created by the drug increases the likelihood that the patient may lose CT into external OR area.

Hypothermia under generalized anaesthesia follows distinct profiles, with early-phase fast drop in CT (Phase I), followed by more gradual decrease in CT (Phases II, III, and IV). A plateau-phase (Phase III) take place on process termination, during which CT stabilises (Figure 4). Thermal redistribution may be responsible for the fast heat loss seen during Phase I in the first hour. Phase II (heat transfer from the warmer perimeter to the rest of the environment) is characterised by a gradual linear decrease that occurs over a period of 2-4 hours, during which thermal loss surpasses metabolic heat generation [39–41]. Phase III (thermal homeostasis) starts following 3 - 4 h, once CTs of 33 to 35 degrees Celsius cause peripheral vasoconstriction [42, 43]. Neuraxial anaesthesia, like generalized anaesthesia, interferes with physiologic thermoregulation, but it does so via a different mechanism. The thresholds for tremors / vasoconstriction are lowered (approximately 0.6°C) with epidural 28,29 and spinal anaesthesia, respectively (1.08°F). Leg skin sensors provide afferent heat input is responsible for a large portion of the control of the CT. Within conventional ORs, constant cold-signals remain generating from peripheral regions, which are then processed [44]. Thermal input, on the other hand, is stopped across the blocked areas in regional anaesthesia. The lack of cold signals that results as a consequence of this is perceived centrally as relative leg warmth, which eventually lowers the shivering and vasoconstriction thresholds. Consequently, a patient who has been regionally anaesthetized may believe that he feels warm while are actually losing heat. Neuraxial anaesthesia is typically combined with sedatives / analgesics, which further compromise regulation by impairing the ability to regulate body temperature[45–48].

### 3.6. Risk Factors

Practitioners would, ideally, detect risk parameters leading to UPH before to performing any surgical operation for improving intra-surgical heat control throughout the process. When it came to identifying risk factors, ASPAN used an evidence-based practise approach[49, 50]. Following the evidence evaluation scale developed by colleagues and Stetler, this method evaluated the strength and quality of proof in descending order[51]. The American College of Cardiology/American Heart Association (ACC/AHA) categories were changed to address risk/benefit ratios, with considerable body of proof confirming such guidelines, and the amount of evidence supporting the recommendations. The following are the definitions for these classes[52]:

  Class I: The benefit exceeds the danger in this case, and the suggestion should be followed through on.

A suggestion falls into Class IIa if the profit exceeds the danger, and it is appropriate to carry out or administer the advise in question.

A suggestion falls into Class IIb if the profit outweighs the risk and it is not irrational to follow or implement the advice.

Classes I, II, and III: The danger exceeds the advantage, therefore the advice would not be carried out or managed.

These suggestions are backed up by three different bodies of proof:

Level-A proof includes proof from several randomised trials / meta-analyses examining various (3–5) populi, having overall reliability in the direction and size of the impact.

A level B proof base would consist of proof from single randomised trials / non-randomized investigations assessing small (2 - 3) population samples.

The proof comes from case-based investigations, treatment quality levels, or skilled opinions containing relatively small (1 - 2) groups.

Unfortunately, neither one of the risk variables found is backed by solid proof, indicating that more study in this area is required. These variables suggest a connection but not necessarily a causal relationship; for example, one patient could carry risk parameters yet not develop hypothermia despite having them. Expectantly, by identifying individuals who are vulnerable to hypothermia during the preoperative evaluation, methods to assist maintain normothermic conditions throughout the peri-surgical phase may be devised.

### 3.7. Perianesthetic Heat Loss

The hypothalamus is in charge of regulating and maintaining body temperature, which is altered during the duration of perianesthesia [53–55]. The effects of generalized and regional anaesthesia on thermoregulation are similar. Generalized anaesthesia impairs the hypothalamus' capacity to control the small margin of temperature variation within which it operates [56, 57]. In turn, this leads in a suppression of both centrally mediated vasoconstriction and peripheral vasodilatation [58, 59]. Regional anaesthesia, on the other hand, causes a centrally mediated vasodilation that prevents peripheral vasoconstriction, resulting in re-distributing core-heat with consequent thermal losses throughout surgical procedure/s [53, 58]. According to research, the majority of patients have predictable patterns of heat loss due to anesthetic-driven thermoregulatory disruption coupled to body contact with colder OR ambient [60, 61]. During anaesthesia, there is a decrease of body heat that happens in 03 stages. During the first hour following operation, Phase I, or redistribution, occurs and anaesthesia due to fast systemic circulatory redistribution from patient core into peripheral areas throughout initial 60 minutes of surgery / anaesthesia. This is indicated through significant CT decrease (1 – 3°C) [58, 59]. In consequent 2 - 3 hours post-surgery, Phase II (linear phase) thermal losses remain, however, CT drops are less drastic/rapid and follows a linear trend. A decrease in the rate of decrease in the patient CT is caused by thermal losses surpassing the amount of heat produced by metabolic processes [58]. Eventually, within Phase III (the plateau-phase), thermostasis is achieved having the least amount of heat loss. When thermal loss matches metabolic heat generation, the body's CT remains constant [58].

The four main processes of thermal loss for operating patients will define the rate of heat loss throughout the linear phase: evaporation, conduction, convection, and radiation. Evaporation routes predominate thermal losses for operating patients.

Radiation, or the transmission of heat from one surface to another despite the presence of a constant ambient temperature, is the most significant source of thermal loss in patients undergoing surgery and anaesthesia. When it comes to heat loss in this population, convection is the second most frequent culprit. Conduction and convection both use heat transmission mechanisms that are quite similar. During surgery, the evaporation of physiological fluids during breathing offers an additional pathway for the loss of core body temperature (Figure 5).

### 3.8. Physiological Changes as a Result of Hypothermia

An association linked between hypothermia and the myriad of physiological effects that occur as a consequence of anaesthesia, and this connection is well established (Figure 6). The physiological consequences are characterised by a generalized slowing of metabolism that affects all bodily systems [58, 62, 63]. Apart from the physiological consequences of hypothermia, other possibly harmful consequences include myocardial infarction, impaired wound healing, coagulopathy, improved contagion rates and prolonged advent from anaesthesia due to reduced drug metabolism along with psychological consequences such as stress, pain and changed cognitive functioning [62]. However, while all patients are at increased risk of developing adverse physiological changes as a result of hypothermia, burns and trauma, senior and disabled, infants, mal-nourished patients are among those who are most likely to experience physiological changes as a result of the condition [56]. One study looking at prognostic variables in hypothermia identified patients >70 years had higher risks for adverse consequences linked to improvement of peri-surgical hypothermia [64].

### 3.9. Peri-surgical Hypothermia and Its Risk Factors

Many variables lead to the improvement of peri-surgical hypothermia, some of which are listed below. In accordance with current study and previous research, aetiology / connection of variables involved with accidental hypothermia are well understood and supported. Temperature and timing of the room natural light are critical. The ambient room temperature continues to be the most important interoperative variable in determining whether or not patients will develop hypothermic during surgery. In three landmark investigations, researchers discovered that all patients who entered operating rooms with external temperatures <70°F (21°C) were hypothermic [65–67]. As part of the research, there were no intra-surgical warming treatments given to the patients in this group. The findings revealed that the largest CT drops occurred within initial 60 minutes of presence inside OR [67]. This body of classic research, dating to 1960s - 1970s, provides substantial proof in support of regulating the ambient temperature aimed at preserving thermostasis across surgery cases. Despite this, present operating rooms remain chilly. Adjusting the operating room thermostat to 70°F (21°C) as soon as the patient enters OR could reduce risk of accidental hypothermia occurring. 18 Additional comfort will be provided by maintaining the patient swaddled as best-possible, as well as by decreasing thermal loss [68].

### 3.10. Anaesthetic Technique

Local and generalized anaesthesia both lead to the loss of body temperature in surgical patients by redistributing heat away from the body's centre and toward the periphery, respectively [69, 70]. Regional anaesthesia, on the other hand, causes heat loss mostly as a result of peripheral nerve block, rather than the change of the hypothalamus controlling centre for temperature regulation that happens with generalized anaesthesia [58]. Regional anaesthetic impairs the patient's capacity to constrict his or her blood vessels. When it comes to spinal and epidural anaesthesia, the legs are the primary organs responsible for the transfer of body heat. The use of generalized anaesthesia in conjunction with local anaesthetic allows for the maximum degree of heat loss in operating patients [53]. Understanding the kind of anaesthetic, a patient has had will assist the peri-surgical nurse and the perianesthesia team in developing a complete plan of care to maintain normothermia in the patient.

### 3.11. Hypothermia and Its Consequences

The goal of reducing peri-surgical hypothermia needs a collaborative effort all over the surgical process. When it comes to maintaining proper thermal balance in surgery patients, awareness and training of the whole operating team, containing preoperative, intra-surgical, and post-operative nurses as well as anaesthetic providers, surgeons, and surgery technicians, are essential. The frequency of this avoidable illness will continue to rise unless efforts are made to educate all physicians who deal with operating patients before, during, and after surgical treatment about hypothermia and its potentially life-threatening consequences. The American Society of Plastic Surgeons (ASPAN) has well defined guidelines for avoiding hypothermia in surgery patients [71]. but, research aiming at demonstrating a link between these recommendations and a reduction in the prevalence of hypothermia has been difficult to conduct.

Preoperative some patients come in the operating room with hypothermia, but there is no information available on the prevalence of preoperative hypothermia. Showers in the morning, skin preparations, scant-clothing, together with vasodilator impact from pre-medication form variables that lead to a drop in body temperature. Preoperatively, one of the most essential goals should be to get the patient to surgery in a state of normal thermal balance. As a result, maintaining patients warm before entering the operating room highlights the requirement of early nurse involvement targeted at preserving normothermia in the patient [72, 73]. In order to maintain preoperative normothermia, blankets and forced-air warming equipment may be used, which could aid lower prevalence of peri-surgical hypothermia. Moreover, warming patients before they enter the operating room has been shown to have anxiolytic effects and to make the insertion of intravenous catheters easier [74]. In addition to caps and warming lights, which may be beneficial for babies, there is a paucity of research on their effectiveness.

### 3.12. Intra-surgical

Hypothermia during surgery may be substantially reduced if the operating room temperature is maintained at 70°F throughout the procedure [75, 76]. Although 70°F may appear excessively warm to the operating room personnel, maintain the environment warm until the incision could help to substantially minimise the first Phase I drop in body temperature after the incision. Warming blood products, IV fluids and irrigants may all help to keep the body's thermal balance in normal range. Anesthetic gases that have been heated and humidified also have a role an essential function in maintaining body temperature. Additionally, the use of warming blankets, layered draperies, and head coverings may help to offer extra thermal protection. Forcible warming has been shown to be one of the most efficient treatments for sustaining intra-surgical hypothermia, according to research [77]. The use of forcible heating equipment in the operating room helps to reduce radiant heat loss, which helps to keep the patient's body temperature stable [77].

## 4. Conclusion

Temperature regulation during the time of anaesthesia and peri-surgical care is affected by a variety of factors, and maintaining control over these factors is frequently challenging. When it comes to patient care, having a strong theoretical foundation is essential. Understanding the temperature physiology regulation and the risk factors linked with accidental hypothermia are important to have. Clearly, the body temperature of all operating patients, particularly those who are at risk of emerging hypothermia, must be closely monitored. The perianesthesia/peri-surgical team is in charge of putting in place preventative measures to keep the patient's body temperature as low as possible. According to the most recent research, rather than relying on a single preventative technique to reduce heat loss in the postoperative patient, it is essential to combine several methods for optimizing endpoints. In order to extend and support current data on treatments regarded most effective for reducing the prevalence of hypothermia all over the perianesthesia/peri-surgical cycle, further research is required. For example, research into preoperative treatments to guarantee that patients enter the operating room in near-normal thermal balance provides a chance to link the gap between research and practise in today's peri-surgical and anaesthetic settings. To use ideal proof to improve heat balance in the surgical patient necessitates the use of current and new investigation results throughout the whole perianesthesia/peri-surgical phase, which includes the full surgical procedure.

## Figures and Tables

**Figure 1:** AORN Guideline for Prevention of Unplanned Patient Hypothermia. In briefly, peri-surgical registered nurse must conduct pre-surgical nursing assessment for ruling out risk factor manifestations driving unintentional hypothermia. Throughout peri-surgical period, the peri-surgical group must take and track patient thermal readings. The peri-surgical team should take preventative measures to avoid unintentional hypothermia.

**Figure 2:** Neonatal physiological dysfunctions linked to hypothermia.

**Figure 3:** CT/heat re-distribution throughout generalized anaesthesia.

**Figure 4:** Typical thermal shift profiles observed during generalized anaesthesia. Reproduced with permission from [32].

**Figure 5:** Balance between thermolysis and thermogenesis.

**Figure 6:** A model of thermoregulatory control.

## Data Availability

Data will be provided upon the corresponding author request.

## References

[1] Morris R. H. (1971). Operating room temperature and the anesthetized, paralyzed patient. *Archives of Surgery*.

[2] Kurz A. (2008). Physiology of thermoregulation. *Best Practice & Research Clinical Anaesthesiology*.

[3] Frank S. M. (1997). Perioperative maintenance of normothermia reduces the incidence of morbid cardiac events. *JAMA*.

[4] Blondin N. A. (2014). Diagnosis and management of periodic hypothermia. *Neurology: Clinical Practice*.

[5] Zagkle E., Grosiak M., Bauchinger U., Sadowska E. T. (2020). Rest-phase hypothermia reveals a link between aging and oxidative stress: a novel hypothesis. *Frontiers in Physiology*.

[6] Tjoakarfa C., David V., Ko A., Hau R. (2017). Reflective blankets are as effective as forced air warmers in maintaining patient normothermia during hip and knee arthroplasty surgery. *The Journal of Arthroplasty*.

[7] Koc B. B., Schotanus M. G. M., Kollenburg J.-P. A. P. A. C., Janssen M. J. A., Tijssen F., Jansen E. J. P. (2017). Effectiveness of early warming with self-warming blankets on postoperative hypothermia in total hip and knee arthroplasty. *Orthopaedic Nursing*.

[8] Noll E., Diemunsch S., Pottecher J. (2018). Prevention of laparoscopic surgery induced hypothermia with warmed humidified insufflation: is the experimental combination of a warming blanket synergistic?. *PLoS One*.

[9] Shimaoka H., Shiina T., Suzuki H., Horii Y., Horii K., Shimizu Y. (2021). Successful induction of deep hypothermia by isoflurane anesthesia and cooling in a non-hibernator, the rat. *The Journal of Physiological Sciences*.

[10] Shimaoka H., Kawaguchi T., Morikawa K. (2018). Induction of hibernation-like hypothermia by central activation of the A1 adenosine receptor in a non-hibernator, the rat. *The Journal of Physiological Sciences*.

[11] Li C., Zhao B., Li L., Na G., Lin C. (2021). Analysis of the risk factors for the onset of postoperative hypothermia in the postanesthesia care unit. *Journal of Perianesthesia Nursing: Official Journal of the American Society of PeriAnesthesia Nurses*.

[12] Yitayew Y. A., Aitaye E. B., Lechissa H. W., Gebeyehu L. O. (2020). Neonatal hypothermia and associated factors among newborns admitted in the neonatal intensive care unit of dessie referral hospital, amhara region, northeast Ethiopia. *International Journal of Pediatrics*.

[13] Liu M., Qi L. (2021). The related factors and countermeasures of hypothermia in patients during the anesthesia recovery period. *American Journal of Tourism Research*.

[14] Bindu B., Bindra A., Rath G. (2017). Temperature management under generalized anesthesia: compulsion or option. *Journal of Anaesthesiology, Clinical Pharmacology*.

[15] Card E. B., Wells N., Mesko P., Eliades A., MacDonald R., Krenzischek D. A. (2021). Perianesthesia nurses pain management practices: findings and recommendations from a national descriptive study of members of the American society of perianesthesia nurses. *Journal of PeriAnesthesia Nursing*.

[16] Osilla E. V., Marsidi J. L., Sharma S. (2021). *Physiology, Temperature Regulation*.

[17] Oguz F., Yildiz I., Varkal M. A. (2018). Axillary and tympanic temperature measurement in children and normal values for ages. *Pediatric Emergency Care*.

[18] Kalasbail P., Makarova N., Garrett F., Sessler D. I. (2018). Heating and cooling rates with an esophageal heat exchange system. *Anesthesia & Analgesia*.

[19] Madrid E. (2016). Active body surface warming systems for preventing complications caused by inadvertent peri-surgical hypothermia in adults. *Cochrane Database of Systematic Reviews*.

[20] House C. M., Tipton M. J., Hopkins P. M., Roiz de Sa D. (2019). Thermoregulation and markers of muscle breakdown in malignant hyperthermia susceptible volunteers during an acute heat tolerance test. *Journal of Science and Medicine in Sport*.

[21] Gauer R., Meyers B. K. (2019). Heat-related illnesses. *American Family Physician*.

[22] Pumchandh N. (2012). Monitoring of the bed time body temperature and body weight to prevent the occurrence of heat stroke in the Royal Thai Army recruits, Lopburi Province, Thailand. *Medical Journal of the Medical Association of Thailand*.

[23] Xu L., Tao Z.-Y., Lu J.-Y. (2019). A single-center, prospective, randomized clinical trial to investigate the optimal removal time of the urinary catheter after laparoscopic anterior resection of the rectum: study protocol for a randomized controlled trial. *Trials*.

[24] Boisson M., Alaux A., Kerforne T. (2018). Intra-operative cutaneous temperature monitoring with zero-heat-flux technique (3M SpotOn) in comparison with oesophageal and arterial temperature. *European Journal of Anaesthesiology*.

[25] Bayraktar S., Balcı S., Ince Z. (2021). The effect of 2 humidifier temperature settings on inspired gas temperatures and the physiological parameters of preterm infants receiving mechanical ventilation therapy. *Advances in Neonatal Care*.

[26] Magoon R. (2020). Precision cardiac anesthesia: welcome aboard!. *Journal of Cardiothoracic and Vascular Anesthesia*.

[27] Daniels J., Kulstad E. (2021). Further mechanistic evidence against luminal esophageal temperature monitoring?. *Journal of Cardiovascular Electrophysiology*.

[28] Alhammoud M., Oksa J., Morel B., Hansen C., Chastan D., Racinais S. (2021). Thermoregulation and shivering responses in elite alpine skiers. *European Journal of Sport Science*.

[29] Kim H., Kim S., Lee M. (2021). Smart patch for skin temperature: preliminary study to evaluate psychometrics and feasibility. *Sensors*.

[30] Oliveira P. E. A., Salvador G. H. M., Marchi-Salvador D. P. (2020). Malignant hyperthermia in bariatric surgery: a case study with clinical, pathophysiological, biochemical and biophysical correlations. *Journal of Medical Cases*.

[31] Bashaw M. A. (2016). Guideline implementation: preventing hypothermia. *AORN Journal*.

[32] Miller R. D. (2010). *Miller’s Anesthesia*.

[33] Matsukawa T., Sessler D. I., Sessler A. M. (1995). Heat flow and distribution during induction of general anesthesia. *Anesthesiology*.

[34] Chava R., Zviman M., Assis F. R. (2019). Effect of high flow transnasal dry air on core body temperature in intubated human subjects. *Resuscitation*.

[35] Jessen C., Feistkorn G. (1984). Some characteristics of CT signals in the conscious goat. *American Journal of Physiology*.

[36] Columbano N., Duffee L. R., Melosu V. (2018). Determination of minimum alveolar concentration and cardiovascular effects of desflurane in positive-pressure ventilated sheep. *American Journal of Veterinary Research*.

[37] Hem N.-A., Phie J., Chilton L., Kinobe R. (2019). A volume-pressure tail cuff method for hemodynamic parameters: comparison of restraint and light isoflurane anesthesia in normotensive male Lewis rats. *Journal of Pharmacological and Toxicological Methods*.

[38] Rufiange M., Leung V. S. Y., Simpson K., Pang D. S. J. (2020). Pre-warming before general anesthesia with isoflurane delays the onset of hypothermia in rats. *PLoS One*.

[39] Ohki K., Kawano R., Yoshida M., Kanosue I., Yamamoto K. (2019). Normothermia is best achieved by warming above and below with pre-warming adjunct: a comparison of conductive fabric versus forced-air and water. *Surgical Technology International*.

[40] Santos R. (2019). Randomized clinical study comparing active heating methods for prevention of intra-surgical hypothermia in gastroenterology. *Rev Lat Am Enfermagem*.

[41] Thapa H. P., Kerton A. J., Peyton P. J. (2019). Comparison of the EasyWarm self-heating blanket with the Cocoon forced-air warming blanket in preventing intraoperative hypothermia. *Anaesthesia & Intensive Care*.

[42] Kaiyala K. J., Ramsay D. S. (2018). Concentration-related metabolic rate and behavioral thermoregulatory adaptations to serial administrations of nitrous oxide in rats. *PLoS One*.

[43] Cobb B., Cho Y., Hilton G., Ting V., Carvalho B. (2016). Active warming utilizing combined IV fluid and forced-air warming decreases hypothermia and improves maternal comfort during cesarean delivery. *Anesthesia & Analgesia*.

[44] Rajek A., Greif R., Sessler D. I. (2001). Effects of epidural anesthesia on thermal sensation. *Regional Anesthesia and Pain Medicine*.

[45] Matsukawa T., Kurz A., Sessler D. I., Bjorksten A. R., Merrifield B., Cheng C. (1995). Propofol linearly reduces the vasoconstriction and shivering thresholds. *Anesthesiology*.

[46] Kurz A., Go J. C., Sessler D. I., Kaer K., Larson M. D., Bjorksten A. R. (1995). Alfentanil slightly increases the sweating threshold and markedly reduces the vasoconstriction and shivering thresholds. *Anesthesiology*.

[47] Taylor N. A. S., Nykvist Å, Powers N., Caldwell J. N. (2019). Thermoeffector threshold plasticity: the impact of thermal pre-conditioning on sudomotor, cutaneous vasomotor and thermogenic thresholds. *Journal of Thermal Biology*.

[48] Lenhardt R. (2018). Body temperature regulation and anesthesia. *Thermoregulation: From Basic Neuroscience to Clinical Neurology, Part II*.

[49] Hooper V. D., Chard R., Clifford T. (2009). ASPAN’s evidence-based clinical practice guideline for the promotion of perioperative normothermia. *Journal of PeriAnesthesia Nursing*.

[50] Lepkowski A. M., Maughan E. D. (2018). Introducing NASN’s new evidence-based clinical guideline: students with seizures and epilepsy. *NASN School Nurse*.

[51] Stetler C. B. (1998). Proof-based practice and the role of nursing leadership. *The Journal of Nursing Administration*.

[52] Eagle K. A. (1996). Guidelines for peri-surgical cardiovascular evaluation for noncardiac surgery. Report of the American College of Cardiology/American heart association task force on practice guidelines (committee on peri-surgical cardiovascular evaluation for noncardiac surgery). *Journal of the American College of Cardiology*.

[53] Kiekkas P., Karga M. (2005). Prewarming: preventing intraoperative hypothermia. *British Journal of Perioperative Nursing*.

[54] Good K. K., Verble J. A., Secrest J., Norwood B. R. (2006). Postoperative hypothermia-The chilling consequences. *AORN Journal*.

[55] Weirich T. L. (2008). Hypothermia/warming protocols: why are they not widely used in the OR?. *AORN Journal*.

[56] Tander B., Baris S., Karakaya D., Ariturk E., Rizalar R., Bernay F. (2005). Risk factors influencing inadvertent hypothermia in infants and neonates during anesthesia. *Pediatric Anesthesia*.

[57] Lewden A., Nord A., Bonnet B., Chauvet F., Ancel A., McCafferty D. J. (2020). Body surface rewarming in fully and partially hypothermic king penguins. *Journal of Comparative Physiology B*.

[58] Sessler D. I., Todd M. M. (2000). Perioperative heat balance. *Anesthesiology*.

[59] Taguchi A., Kurz A. (2005). Thermal management of the patient: where does the patient lose and/or gain temperature?. *Current Opinion in Anaesthesiology*.

[60] Koh W., Chakravarthy M., Simon E. (2021). Perioperative temperature management: a survey of 6 Asia-Pacific countries. *BMC Anesthesiology*.

[61] Ingram A., Harper M. (2018). The health economic benefits of perioperative patient warming for prevention of blood loss and transfusion requirements as a consequence of inadvertent perioperative hypothermia. *Journal of Perioperative Practice*.

[62] Ayres U. (2004). Older people and hypothermia: the role of the anaesthetic nurse. *British Journal of Nursing*.

[63] Buhre W., Rossaint R. (2003). Perioperative management and monitoring in anaesthesia. *The Lancet*.

[64] Kongsayreepong S., Chaibundit C., Chadpaibool J. (2003). Predictor of core hypothermia and the surgical intensive care unit. *Anesthesia & Analgesia*.

[65] Kumar S., Wong P. F., Melling A. C., Leaper D. J. (2005). Effects of perioperative hypothermia and warming in surgical practice. *International Wound Journal*.

[66] Morris R. H., Wilkey B. R. (1970). The effects of ambient temperature on patient temperature during surgery not involving body cavities. *Anesthesiology*.

[67] Goldberg M. J., Roe C. F. (1966). Temperature changes during anesthesia and operations. *Archives of Surgery*.

[68] Pich J. (2020). Intravenous nutrients for preventing inadvertent peri-surgical hypothermia in adults. *Journal of Perioperative Practice*.

[69] Alfonsi P., Bekka S., Aegerter P. (2019). Prevalence of hypothermia on admission to recovery room remains high despite a large use of forced-air warming devices: findings of a non-randomized observational multicenter and pragmatic study on perioperative hypothermia prevalence in France. *PLoS One*.

[70] Li Y., Liang H., Feng Y. (2020). Prevalence and multivariable factors associated with inadvertent intraoperative hypothermia in video-assisted thoracoscopic surgery: a single-center retrospective study. *BMC Anesthesiology*.

[71] Burns S. M., Wojnakowski M., Piotrowski K., Caraffa G. (2009). Unintentional hypothermia: implications for perianesthesia nurses. *Journal of PeriAnesthesia Nursing*.

[72] Wagner V. D. (2006). Unplanned perioperative hypothermia. *AORN Journal*.

[73] Croke L. (2019). Guideline for prevention of hypothermia. *AORN Journal*.

[74] Xu H., Wang Z., Guan X. (2020). Safety of intraoperative hypothermia for patients: meta-analyses of randomized controlled trials and observational studies. *BMC Anesthesiology*.

[75] Collins S., Budds M., Raines C., Hooper V. (2019). Risk factors for perioperative hypothermia: a literature review. *Journal of PeriAnesthesia Nursing*.

[76] Honkavuo L., Loe S. A. K. (2020). Nurse anesthetists’ and operating theater nurses’ experiences with inadvertent hypothermia in clinical perioperative nursing care. *Journal of PeriAnesthesia Nursing*.

[77] Cooper S. (2006). The effect of preoperative warming on patients’ postoperative temperatures. *AORN Journal*.

